# Prognostic Value of Procalcitonin for Morbidity and Mortality in Patients after Cardiac Surgery

**DOI:** 10.1155/2021/1542551

**Published:** 2021-07-26

**Authors:** Ahmad Amouzeshi, Farshid Abedi, Mahmoud Zardast, Yaser Rezaeian Bilondi, Zahra Amouzeshi

**Affiliations:** ^1^Department of Cardiovascular Surgery, Cardiovascular Diseases Research Center, Birjand University of Medical Sciences, Birjand, Iran; ^2^Birjand University of Medical Sciences, Birjand, Iran; ^3^School of Medicine, Medical Toxicology and Drug Abuse Research Center, Birjand University of Medical Sciences, Birjand, Iran; ^4^Birjand University of Medical Sciences, Birjand, Iran; ^5^Faculty of Nursing and Midwifery, Cardiovascular Diseases Research Center, Birjand University of Medical Sciences, Birjand, Iran; ^6^Isfahan University of Medical Sciences, Isfahan, Iran

## Abstract

**Background:**

The increased serum procalcitonin (PCT) level in cardiac patients is known as a sign of postoperative complications.

**Objective:**

Considering the importance of predicting the incidence of both complications and mortality caused by coronary artery bypass graft (CABG) surgery, this study was conducted to determine the serum PCT level and its relationship with one-year morbidity and mortality among CABG patients.

**Methods:**

This descriptive-analytical study was performed on 100 patients who underwent CABG surgery in Vali-e-Asr Hospital of Birjand, Iran. They were selected by a census sampling method from March 2014 to March 2015. The Elecsys BRAHMS PCT kit (Roche Company) was then used to measure the patients' serum PCT level. The required data were collected using the patients' medical records and telephone interviews with the patient or his/her relatives by passing one year from their discharge. The outcomes of this study comprised of mortality and morbidity causes (e.g., dysrhythmia, infection, and stroke). The data were then analyzed in SPSS version 16 by Mann–Whitney, chi-squared, and Fisher exact tests.

**Results:**

The postoperative serum PCT level is significantly correlated with sternum wound infection (*p*=0.001), packed cells (PC) transfusion (*p*=0.003), and death (*p*=0.003). In addition, a significant relationship was found between dyslipidemia and hypertension and early mortality rate in patients with high levels of PCT. Of note, risk-adjusted death did not differ significantly between the serum PCT levels after one year (RR, 0.068; 95% CI 0.008–0.566).

**Conclusion:**

Higher PCT serum levels in CABG patients are associated with the increased early mortality rate, sternum wound infection, and PC transfusion. Additionally, the other factors associated with mortality in the patients under study included dyslipidemia and hypertension.

## 1. Introduction

High levels of procalcitonin (PCT) are associated with various conditions causing systemic inflammation and their severity, including severe burns, trauma, extensive surgeries, especially cardiac surgery with cardiopulmonary bypass, postresuscitation syndrome, acute pancreatitis, stroke, acute graft rejection, and subarachnoid hemorrhage [1, 2].

The peak level of PCT was observed to be related to various types of surgery such as thoracic, orthopedic, and oncological surgeries [3–6]. Moreover, it is currently well known that the increased serum PCT is an independent predictor of all causes of in-hospital mortality in patients intensive care units (ICU) and is also correlated with poor outcomes after cardiac surgery. PCT is a recognized marker occurring after elective cardiac surgery. The increased serum PCT level in cardiac patients is known as a sign of postoperative complication [5]. Previous studies in this regard have shown a correlation among high levels of postoperative PCT and mortality, infection, and other severe postcardiac surgery complications [7]. Correspondingly, the results of a prospective cohort study conducted by Klingele et al. [5] on patients with cardiac surgery showed that the increased PCT levels after surgery could be regarded as a prognostic indicator for both infection and postoperative complications. As well, single measurements of postoperative PCT levels could predict the delayed complications among elective cardiac surgery patients, despite a postoperative period without any significant event. Identifying such people at risk before being discharged from the ICU can prevent readmission and also ensure appropriate monitoring and rapid treatment of emerging complications.

The PCT algorithm, which is examined to decide on the antibiotic treatment of adult patients admitted to primary care, emergency care, and ICU, suggests that performing the treatment guided by PCT may consequently reduce the exposure to antibiotics without increasing the mortality rate [8].

Therefore, given the importance of predicting the incidence of both complications and mortality caused by CABG surgery, this study was conducted to determine the serum PCT level and its relationship with early morbidity and mortality among CABG patients.

## 2. Materials and Methods

This descriptive-analytical study was conducted on 100 patients who were hospitalized in the Heart Department of the Vali-e-Asr Hospital in Birjand, Iran. A census sampling method was utilized for including the cases. The inclusion criteria of this study were patients aged between 30 and 80 years old who underwent CABG surgery and admitted to the cardiac department. In addition, the exclusion criteria included concurrent coronary and valve operation, aortic dissection, and pulmonary embolism. The required data were collected using the patient's medical records and telephone interviews with the patient or his/her relatives by passing one year from his/her discharge. The outcomes under scrutiny involved mortality (annual death rate) and morbidity (e.g., dysrhythmia, infection, and CVA). For the purpose of the study, the Elecsys BRAHMS PCT kit (Roche Company) was used to measure the serum PCT level. During the study period, a nurse working in the Cardiac Department collected the blood samples from the included patients before intubation, one hour later in the intensive care unit, and 48 h postoperatively. For examining the serum PCT levels, the obtained samples were stored in due observance of the preservation of the cold chain and then transferred in special kits to Shafa Laboratory of Birjand. The serum PCT level was considered within the normal range of less than or equal to 0.8 ng/ml.

The protocol of the study was approved by the Institutional Ethics Committee with the ID IR.BUMS.REC.1395.236.

Data analysis was performed by SPSS 16 software (IBM Incorporation, Chicago, IL). The normality of quantitative variables was determined using the Kolmogorov–Smirnov test. Besides, categorical variables were analyzed using the chi-square and Fisher exact tests. The Mann–Whitney test was also used for comparing continuous variables. We calculated the relative risk (RR) with 95% confidence intervals (CI) to compare the death between serum PCT levels. The significance level was considered less than 0.05.

## 3. Results

The mean age of the patients included in this study was 63.0 ± 10.53 years old, and the majority of them (*n* = 67(67%)) were men. The demographic and medical characteristics of these 100 patients are given in Table 1. The mean score ±standard deviation of the serum PCT levels of the patients before, immediately after, and 48 hours after surgery were obtained as 0.05 ± 0.06, 0.08 ± 0.11, and 1.44 ± 3.06, respectively. The results of the present study show a significant relationship among postoperative serum PCT level and sternum wound infection (*p*=0.001), PC transfusion (*p*=0.003), and death (*p*=0.003). However, no significant association was found between the serum PCT level and the incidence of both dysrhythmia and EF (*p* > 0.05) (Table 2). The results also show that a significant relationship exists among dyslipidemia, hypertension, and early mortality rate in patients with high levels of PCT (Table 3).

After the one-year follow-up, of the nine deaths in this study, one case of death occurred during surgery and seven cases occurred in the hospital ward. By passing 30 days from their discharge, one case of death was reported as well. Therefore, mortality is considered as “Early mortality.” These deaths were resulted from all causes of mortality, consisting of three patients (33.33%) due to cardiac causes, one case (11.11%) from brain causes, two cases (22.22%) from renal causes, one case (11.11%) from heart attack, and eventually two cases (22.22%) due to unknown reasons.

During this one-year follow-up, except for those listed as early morbidity, no other case was reported. Hence, morbidity is considered as early morbidity.

Risk-adjusted death showed a significant relationship with the serum PCT levels after one year (RR, 0.068; 95% CI 0.008–0.566).

## 4. Discussion

This study aimed to determine how the serum PCT level is associated with both early morbidity and mortality among CABG patients. The results show that serum PCT levels in the patients before, after, and 48 hours after surgery were 0.05 ± 0.06, 0.08 ± 0.11, and 1.44 ± 3.06, respectively, indicating an increase in this inflammatory marker rate after performing the surgery. A study by Arkader et al. [9] on patients who underwent cardiopulmonary bypass (CPB) showed that the PCT baseline level increased after CPB and peaked at 24 hours, which was consistent with the results of the present study.

The results of the present study reveal that those receiving over two units of PC during the treatment and surgery had a significantly higher PCT level compared to those receiving smaller PC quantities. The results of several previous studies have demonstrated that the increased PC transfused during surgery is associated with postoperative complications and higher rates of mortality and morbidity after surgery [10–12]. Additionally, some studies have previously shown that the rise in the PCT level among patients undergoing CABG is associated with the increased consequent complications [5, 13, 14]. Therefore, the results obtained in the present study are in line with those of previous studies where the increased transfused PC along with higher levels of PCT can be considered as useful markers for a higher number of complications after surgery.

Based on the results of the present study, there was a significant relationship between the PCT level and some factors such as wound infection. Previously, the results of various studies have shown that inflammation is an arrhythmic stimulant, and the increased PCT levels are associated with the increased inflammation and postoperative complications [13–17]. For example, the results of a study by Klingele et al. [5] have shown that the increased postoperative PCT level is a prognostic marker for both infection and complications, which were consistent with the results of the present study.

The results of the present study show that the increased PCT level is significantly associated with an increase in the early mortality rate. Moreover, Dorge et al. [14] in their studies have shown that the survival rate is lower in patients with high levels of serum PCT in the first 24-hour postoperatively. Another study have also reported that the PCT level >2.5 ng·l (−1) can be regarded as a predictor for mortality within the first 28-day of CABG surgery [18].

Besides, the results indicate a significant relationship between early mortality rate and dyslipidemia in the patients with high PCT levels. However, some ambiguities still exist regarding the role of low blood lipids in the outcome of cardiovascular surgery. In the study by Hosseini and Mehrpooya [19], the mean TG, LDL, and HDL levels were not significantly correlated with mortality rate. However, there was a significant difference in terms of the in-hospital mortality between patients with the controlled and noncontrolled LDL, HDL, and TG levels. A meta-analysis has also shown that preoperative statin therapy could reduce the mortality rate in patients after cardiac surgery [20]. Nevertheless, Powell et al. [21] in their research have reported that performing lipid-lowering therapy before CABG surgery could not lead to the reduced in-hospital mortality or morbidity (including postoperative atrial fibrillation and hemorrhage). Given the increased risk factors for coronary heart disease along with increased therapeutic costs, it would be a crucial priority to identify and treat risky individuals. Therefore, performing further studies in this area seems to be necessary.

The results of the present study show that a significant relationship exists between hypertension and early mortality rate in patients with high levels of PCT. A prospective population-based study has previously reported a positive association between plasma PCT levels and cardiovascular risk factors such as hypertension, in subjects with no history of acute cardiovascular events [22].

According to the results of the present study, the relationship between diabetes and the incidence of outcomes such as CVA, infection, death, and dysrhythmia for different PCT levels was not statistically significant. The results of the study by Santos et al. [23] showed that although diabetic patients are at high risks of developing complications, diabetes alone cannot be considered as a factor in deteriorating prognosis. Furthermore, the results of the study by Whang and Bigger [24] indicated that diabetes is associated with the increased postoperative complications and rehospitalization, but it is not associated with long-term mortality after CABG surgery among patients with severe left ventricular dysfunction. These results were consistent with the results of the present study. However, the results of Mao's study [25] showed that several factors such as the history of cardiovascular disease, longer duration of operation, postoperative cardiac arrhythmias, and previous carotid artery stenosis in the patients undergoing surgery could increase the risk of postoperative stroke. Accordingly, the difference between the results of the present study and those of previous studies may possibly be due to the number and type of the grafts utilized [26].

Among the limitations of this study were the small sample size and the one-centered setting of the study. Among the other constraints of this research, types of grafts utilized that were not addressed in this study can be named, which limited the generalizability of the results. Therefore, it is recommended that a similar study be performed with a larger sample size in several therapeutic centers, and by focusing on further variables (such as number and type of grafts).

## 5. Conclusion

The increased serum PCT levels in patients underwent CABG surgery are associated with the increased early mortality rate, sternum wound infection, and PC transfusion. Moreover, in our patients, the other factors associated with mortality included dyslipidemia and hypertension.

## Figures and Tables

**Table 1:** The demographic and medical characteristics of the 100 patients participated in the study.

Characteristic		All patients (*n* = 100)
Age, mean ± SD		63.0 ± 10.53

Gender	Male	67 (67)
	Female	33 (33)

Smoker	Yes	13 (13)
	No	87 (87)

No. of grafts, mean ± SD		3.9 ± 0.65

Type of dysrhythmia	No	86 (86)
	VT	6 (6)
	AF	8 (8)

Ejection fraction, %	20–29	12 (12)
	30–39	16 (16)
	40–49	26 (26)
	≥50	46 (46)

DM	Yes	36 (36)
	No	64 (64)

DLP	Yes	46 (46)
	No	54 (54)

HTN	Yes	57 (57)
	No	43 (43)

CVA	Yes	4 (4.0)
	No	96 (96.0)

VT, ventricular tachycardia; AF, atrial fibrillation; DM, diabetes mellitus; DLP, dislipidemia; HTN, hypertension; CVA, cerebrovascular accident.

**Table 2:** Postoperative data and adverse events.

Variable	PCT levels ≤0.8 ng/ml (*n* = 59)	PCT levels >0.8 ng/ml (*n* = 41)	*P* value
Death			0.003
Present	1 (1.7)	8 (19.5)	
Not present	58 (98.3)	33 (80.5)	

Type of dysrhythmia			0.342
Not present	53 (89.8)	33 (80.5)	
VT	2 (3.4)	4 (9.8)	
AF	4 (6.8)	4 (9.8)	

PC			0.003
≤2	37 (63.3)	13 (32.5)	
>2	22 (36.7)	27 (67.5)	

Sternum wound infection			0.001
Present	3 (5.1)	13 (31.7)	
Not present	56 (94.9)	28 (68.3)	

EF (mean ± SD)	45.0 ± 9.74	45.2 ± 9.80	0.98

PC, packed cells; EF, ejection fraction.

**Table 3:** Comparison of the outcomes under scrutiny during a one-year follow-up period based on serum PCT levels and previous diseases.

Variable	Serum PCT level ≤0.8		*P* value	Serum PCT level >0.8		*P* value
	With diabetes, *N* (%)	Without diabetes, *N* (%)		With diabetes, *N* (%)	Without diabetes, *N* (%)	
Dysrhythmia			—			0.765
Yes	0 (0.0)	0 (0.0)		4 (11.4)	10 (16.1)	
No	1 (100.0)	2 (100.0)		31 (88.6)	52 (83.9)	
CVA			—			1.000
Yes	0 (0.0)	0 (0.0)		1 (2.9)	3 (4.8)	
No	1 (100.0)	2 (100.0)		34 (97.1)	59 (95.2)	
Death			—			0.277
Yes	0 (0.0)	0 (0.0)		5 (14.3)	4 (6.5)	
No	1 (100.0)	2 (100.0)		30 (85.7)	58 (93.5)	
Wound infection			—			0.257
Yes	0 (0.0)	0 (0.0)		8 (22.9)	8 (12.9)	
No	1 (100.0)	2 (100.0)		27 (77.1)	54 (87.1)	

Variable	With hypertension, *N* (%)	Without hypertension, *N* (%)	*P* value	With hypertension, *N* (%)	Without hypertension, *N* (%)	*P* value
Dysrhythmia			—			0.569
Yes	0 (0.0)	0 (0.0)		7 (12.5)	7 (17.1)	
No	1 (100.0)	2 (100.0)		49 (87.5)	34 (82.9)	
CVA			—			1.000
Yes	0 (0.0)	0 (0.0)		2 (3.6)	2 (4.9)	
No	1 (100.0)	2 (100.0)		54 (96.4)	39 (95.1)	
Death			—			0.009
Yes	0 (0.0)	0 (0.0)		9 (16.1)	0 (0.0)	
No	1 (100.0)	2 (100.0)		47 (83.9)	41 (100.0)	
Wound infection			—			0.583
Yes	0 (0.0)	0 (0.0)		8 (14.3)	8 (19.5)	
No	1 (100.0)	2 (100.0)		48 (85.7)	33 (80.5)	

Variable	With dyslipidemia, *N* (%)	Without dyslipidemia, *N* (%)	*P* value	With dyslipidemia, *N* (%)	Without dyslipidemia, *N* (%)	*P* value
Dysrhythmia			—			0.018
Yes	0 (0.0)	0 (0.0)		2 (4.5)	12 (22.6)	
No	1 (100.0)	2 (100.0)		42 (95.5)	41 (77.4)	
CVA			—			0.624
Yes	0 (0.0)	0 (0.0)		1 (2.3)	3 (5.7)	
No	1 (100.0)	2 (100.0)		43 (97.7)	50 (94.3)	
Death			—			0.001
Yes	0 (0.0)	0 (0.0)		9 (20.5)	0 (0.0)	
No	1 (100.0)	2 (100.0)		35 (79.5)	53 (100.0)	
Wound infection			—			0.276
Yes	0 (0.0)	0 (0.0)		5 (11.4)	11 (20.8)	
No	1 (100.0)	2 (100.0)		39 (88.6)	42 (79.2)	

## Data Availability

The data used to support the findings of this study are available from the corresponding author upon request.
